# Health Recognition Algorithm for Sports Training Based on Bi-GRU Neural Networks

This article has been retracted.

**DOI:** 10.1155/2021/1579746

**Published:** 2021-07-13

**Authors:** Qi Nie, Yun Li, Wen Ying Xiong, Wei Xu

**Affiliations:** College of Physical Education and Health, Jiangxi University of Traditional Chinese Medicine, Nanchang 330000, China

## Abstract

The healthcare benefits associated with regular physical activity recognition and monitoring have been considered in several research studies. Regular recognition and monitoring of health status can potentially assist in managing and reducing the risk of many diseases such as cardiovascular disease, diabetes, and obesity. Using healthcare equipment in hospitals, people can conduct regular physical examinations to check their health status. However, most of the time, it is difficult to reach a specific medical environment and use special medical equipment. In this paper, a deep learning framework based on the bidirectional gated recurrent unit for health status recognition is implemented to improve the accuracy by making full use of the information provided by smartphone acceleration sensors. A model based on a bidirectional gated recurrent unit is constructed to describe the relationship between input acceleration signals and output information through a gating approach. Therefore, it can automatically detect the health status of the sportsman as healthy, subhealthy, and unhealthy. Finally, the practical data collected from an athlete have been used to evaluate the recognition performance of the system. Results show that the proposed methodology can predicate the sports health status accurately.

## 1. Introduction

During the past decade, the sports health monitoring system (SHMS) [1–4] has attracted much attention from academia and industry. The corresponding research and development efforts have increased year by year. With today's rising healthcare costs [5–8] and the aging world population, athletes must be able to monitor their health status [9] at any time in the context of athletic training, in addition to specific medical settings. Recently, to fulfill this demand, a variety of health monitoring systems are developed. These systems record the user's health status information in real time [10] and then communicate this information to the user or communicate directly to doctors and medical centers. They also alert the users in the case of health problems. In addition, SHMS provides a new approach to the management and monitoring of populations with chronic diseases, the elderly, patients recovering from surgery, children, and people with specific diseases. However, most health monitoring systems [11] have stringent environmental conditions for application. Before collecting and inspecting health-related parameters of the human body, precise and accurate scientific and medical equipment need to be arranged in advance. If they are separated from the specific environment, their performance will be significantly affected. Some technologies even need to be equipped with special computing terminals. The cost of such SHMSs is very high, and there are great technical limitations such as recognition accuracy, computing power, and memory requirement. These problems will greatly limit their promotion and popularization.

Health status recognition [12–15] in sports training has always been a research hotspot in the field of motion and activity recognition. It has a wide range of applications in many fields. In healthcare, it can monitor the health status of the human body to remind people to exercise properly. In military training, it can monitor the movement state of soldiers to reduce the occurrence of injuries and improve the training level. In the case of virtual reality, it can increase the sense of the reality of virtual reality so that users can get a more practical and real experience. In motion state recognition, the usual step is to collect a large number of motion status information and develop a motion state model for motion state recognition. Traditionally, motion state recognition has primarily focused on feature engineering and handcrafted feature. Recently, researchers have focused on deep learning methods [16–18], shifting the prototype from feature extraction to feature learning to improve the classifier's robustness. Without the need to rely on complex, large-scale external equipment based on traditional feature extraction and a special usage environment, this paper [19–22] proposes a sports training health recognition algorithm based on the implicit feature extraction and bidirectional gated recurrent unit (Bi-GRU) neural network. It can measure the level of activity based on the number of steps walked in a period and evaluate the health status of individuals and athletes.

Following are the main contributions of this paper:

1. In this paper, an efficient sports training health status recognition algorithm based on the Bi-GRU neural network is proposed, recognizing the athletes' health status in the training state
2. This paper combines Android and PyTorch technology to transplant a neural network model with better recognition performance and use the smartphone to realize real-time recognition of sports health status

The rest of the paper is organized as follows: Section 2 describes the related work, Section 3 illustrates the proposed methodology of motion state recognition, and Section 4 presents the results. Finally, the conclusion is given in Section 5.

## 2. Related Work

### 2.1. Health Monitoring Based on Walking Motion

A large number of studies have shown that exercise training analysis has proved to be an effective means of health monitoring [23]. Even a simple exercise can also reflect the health status of the athletes, predict the health threats they may face, and provide timely responses and suggestions for treatments. The process of gait deviation from or approaching the normal human gait baseline during exercise can reflect the health status. Observing a patient's walking behavior is the most important part of the neurological examination [24]. The ability to walk has a direct impact on human health and morbidity. As a result, walking is often seen as a primary human daily life activity. In the United States, 30.6 million people over the age of 15 have varying difficulty in performing exercise involving the lower limbs, and 7 million people over the age of 65 have walking disabilities. More than 17 million adults of age 18 and older have severe walking difficulties or are completely unable to walk a quarter of a mile in a row, although $300 million a year is spent on healthcare to treat physical disabilities. In addition to the financial cost, a walking disability can also harm a person's body, leading to complete loss of physical activities in daily life. Lee [25] reported in a recent study that 6–10% of noncommunicable diseases worldwide are caused by insufficient exercise, including coronary artery disease, type II diabetes, breast cancer, and colon cancer, leading to the premature death of 9% of such patients.

### 2.2. Movement Status Recognition

Movement status recognition using smartphone sensors is an important research field full of challenges and opportunities. It is due to the wide range of human activities and the changes in how a particular activity is to be performed. The majority of the studies on movement status recognition focus mainly on accuracy, robustness, and real-time application. Owing to the increased computing and sensing power of the modern smartphone, many healthcare and monitoring application systems are nowadays implemented on smartphones. Modern smartphones are equipped with different types of sensors such as accelerometers, gyroscopes, magnetometers, and proximity sensors. Among these sensors, accelerometer and gyroscope have been widely used for monitoring human activities of daily life and falls due to their lower power requirement and direct capturing of motion data. Foerster et al. [26] used acceleration sensors for human motion state recognition. Bao et al. [27] placed multiple acceleration sensors on different parts of the human body to collect motion state data. They then used a data mining algorithm to analyze the data and classify motion states. With the emergence of human actions and activity recognition, the practice of distributing multiple sensors on various parts of the human body was common. However, with the development of technology, especially with the emergence of smartphones with embedded miniature sensors, researchers prefer to use smartphones to replace the traditional data collection method. Kwapisz et al. [28] used the acceleration sensor embedded in smartphones to collect motion data and found that the position and orientation of the sensors had a great impact on the performance of the motion recognition. The sensor's signals were preprocessed, and discriminant features were extracted from the processed signals. However, during classification, the classifier was unable to classify more similar motion states accurately.

Generally, the performance of motion state recognition systems depends on the type of sensor being used, the data acquisition method, the preprocessing approach, the feature extraction algorithm, and the type of classifier. In order to improve the recognition performance of the classifier, researchers have developed novel preprocessing and feature extraction methods. Jiang and Yin [29] conducted secondary processing on the collected sensor's data to convert the signal data into image information. In this process, the collected sensor signals were arranged and represented as image data. Then, these image data were input into a deep convolutional neural network for feature extraction and recognition. The classification results on different image data were then compared. Ronao and Cho [30] also applied a deep convolutional neural network (CNN) for automatic feature learning. They provided a method to extract robust data features from the original data automatically. Experimental results showed that each layer of CNN can still distinguish complex features, although the complexity level of each layer of features decreases. Shafique and Hato [31] used acceleration sensors to identify human traffic conditions and mainly discussed data preprocessing, methods of selecting and generating training data, and classifier selection. Four different classification algorithms, such as support vector machine (SVM), AdaBoost, decision tree (DT), and random forest (RF), were used for classification, and the results were analyzed. However, the main limitation of their work was the application of special equipment to collect data, which will undoubtedly cause new problems for the broad application of equipment in the future.

## 3. Methodology

For the recognition of sports training health status, this article mainly studies two aspects of human motion. One is to recognize the human motion state. We use the motion posture estimation method. The data are mainly collected in the indoor environment; the other is developing a model based on the human motion state. This article mainly collects human activities' data through smartphone acceleration sensors such as accelerometer and gyroscope and develops a health status recognition model based on the Bi-GRU neural network model that can be implemented in smartphones. This process involved data collection, preprocessing, data format conversion, neural network model construction, parameter adjustment, training the model, and testing the model.

### 3.1. Motion Pose Estimation

In this paper, based on the quaternion attitude estimation algorithm, the attitude angle can be obtained by integrating the data value measured by the gyroscope sensor over time. Whenever the quaternion is updated with the latest gyroscope measurement value, the attitude angle can be calculated by the following formula:

(1) $$\begin{array}{c} \left\{\begin{array}{c} \phi =\arctan\;2\left(2\left(q_{0}q_{1}+q_{2}q_{3}\right)\right.,\;1-2\left(q_{1}^{2}+q_{2}^{2}\right),\\ \theta =\arcsin\left(2\left(q_{0}q_{2}-q_{1}q_{3}\right)\right),\\ \psi =\arctan\;2\left(2\left(q_{0}q_{3}+q_{1}q_{2}\right),\;1-2\left(q_{2}^{2}+q_{3}^{3}\right)\right)-D, \end{array}\right. \end{array}$$

where *D* is the declination angle of the geomagnetic field.

Under normal circumstances, the athlete's gait is periodic and regular, and each walking cycle is composed of a series of ordered gait events and related gait phases such as swing and stance phases. Based on the above information, we can use the sensor to realize gait detection. Since the gait movement mainly occurs in the sagittal plane, the gait event detection can be distinguished by the rotation state of the thigh in this plane. Therefore, a gait event detection method based on thigh angle is proposed in this paper.

As shown in Figure 1, the thigh angle *γ* is defined as the angle of the thigh from the vertical direction. It can be seen from the figure that although *θ*=*γ* exists (they are the complementary angles of the same angle), the thigh angle *γ* reflects the thigh swing phase more obviously than the pitch angle *θ* (*θ* refers to the angle of rotation around the *X*-axis from the horizontal direction). Generally speaking, the sign of the angle *γ* depends on the rotation direction of the thigh. When the thigh is approximately parallel to the vertical axis of gyroscopes, *γ*=0; when the thigh rotates counterclockwise around the positive semiaxis of *X*, *γ* > 0; when the thigh rotates around *X* when the positive semiaxis rotates clockwise, *γ* < 0.

### 3.2. GRU and Bi-GRU Neural Network

A recurrent neural network (RNN) is a kind of artificial neural network with a memory function suitable for sequence data modeling. However, typical RNNs face the issues of gradient explosion and gradient disappearance, and these cannot grip long-distance dependence problems. For this reason, Hochreiter and Schmidhuber [32] proposed a long short-term memory (LSTM) neural network, a special RNN that performs better on longer sequences. Chao et al. [33] proposed the GRU neural network based on LSTM neural networks. They combined the forget gate and input gate in an LSTM neural network into a single “update gate” and combined the cell state and hidden state. The GRU neural network is a circular network structure that determines the current output information through the input information at the current moment and the output information at the last moment. Therefore, the output information at each moment in the GRU neural network depends on past information. Therefore, its chain attribute is closely related to the sequential labeling problem. The unit structure of the GRU is shown in Figure 2.

The process of obtaining a linear sum between the existing state and the newly computed state is similar to that of an LSTM cell. However, GRU does not have any mechanism to control the exposure level of its state, showing the entire state each time. The calculation equation of the GRU is as follows:

(2) $$\begin{array}{c} z_{t}=\sigma \left(w_{z}\times \left[h_{t-1},x_{t}\right]\right),\\ r_{t}=\sigma \left(w_{\text{r}}\times \left[h_{t-1},x_{t}\right]\right),\\ {\tilde{h}}_{t}=\text{tan}h\left(w\times \left[r_{\text{t}}*h_{t-1},x_{t}\right]\right),\\ h_{t}=\left(1-z_{t}\right)*h_{t-1}+z_{t}*h_{t}, \end{array}$$

where *x*, *h*, *z*, and *r* are the input vector, output vector, update gate state, and reset gate state, respectively, and *W* is the parameter matrix. Moreover, *h*_*t*_ corresponds with weight matrices and denotes that the candidate activation is based on the previous state and current input. Finally, the output of the hidden unit includes the update part and the previous part. *σ* represents the activation function which ranges from 0 to 1. Activation functions are important features of a neural network and decide to activate or ignore a node based on the relevancy of information received by a node.

After extracting the features using the BI-GRU neural network, the next step is to classify the data. This article uses a softmax activation function to process the value of the output. The softmax activation function was implemented at the output layers to make the final decision for the multiclass classification. Its calculation equation is as follows:

(3) $$\begin{array}{c} P=\arg\max_{c}p\left(y=c|x\right)\\ =\arg\max_{c}\frac{\text{exp}\left({\text{output}}_{t}\right)}{\sum_{k=1}^{K}{\text{output}}_{t}}, \end{array}$$

where *c* is the class label, *x* is the sample feature, *y* is the label variable, *K* is the total number of classes, and output_*t*_ is the output of each layer. It can be seen that softmax classification is a classification result based on probability. The final result of softmax is the probability of identifying certain data as each class in the current data, and the sum of the probability of the classification result for a piece of data is 1.

In establishing the neural network model, it is necessary to consider the occurrence of data overfitting. This article uses regularization to prevent the occurrence of data overfitting. Its idea is to add a new indicator to the loss function to describe the complexity of the model. There are two types of regular expressions: *L*1 and *L*2 regular expressions. The calculated equations are as follows:

(4) $$\begin{array}{c} C=C_{0}+\frac{\lambda }{n}\sum_{w}\left|w\right|,\\ C=C_{0}+\frac{\lambda }{2n}\sum_{w}w^{2}, \end{array}$$

where *C*_0_ is the loss function, *λ* is the proportion of the model's complexity loss in the total loss, and ∑|*w*|∑*w*^2^ describes the complexity of the model. Regardless of the regularization method, the basic idea is to control the size of the weights and suppress the poorly performing weight parameters so that the model cannot randomly fit the wrong feature information. When using *L*1 regularity, the weight is reduced to 0 by a constant, and *L*2 is reduced by an amount proportional to *w*.

Finally, the sports training health recognition model designed in this paper is shown in Figure 3.

## 4. Experiments and Results

This experiment uses the PyTorch0.4 deep learning framework. The Android development platform is Android Studio 3.2. The Python version is 3.6.5, and the graphics card is single GTX3080.

### 4.1. Dataset

In the research process, the public dataset published in [34] and available at https://archive.ics.uci.edu was used. This dataset mainly uses smartphones to collect human movement data. The data contain six actions: walking, walking upstairs, walking downstairs, sitting, standing, and lying. To create the dataset, a group of 30 volunteers followed a protocol of activities while carrying an Android OS-based smartphone attached to a belt on their waist. The dataset comprised 10,299 patterns which were divided into training and test sets in the ratio of 70% to 30%. Each pattern is further represented with a feature vector of 561 elements composed of time and frequency domain features extracted from the accelerometer and gyroscope signals. Accelerometer and gyroscopes are low-powered and low-cost miniature sensors that can measure linear and angular acceleration efficiently. These signals were first preprocessed for noise reduction, and the gravitational component of the acceleration signal was removed. From each window, a vector of features was calculated, including features such as mean, standard deviation, signal magnitude area, interquartile range, autoregression, coefficients, largest fast Fourier transform (FFT) power spectrum component, and correlation coefficients between signal pairs.

### 4.2. Experimental Results

#### 4.2.1. Classification Performance of Different Classifiers

Table 1 summarizes the results obtained with raw acceleration data using different machine learning approaches [35–38]. It can be observed that, after 200 tests, the classification performance of the BI-GRU neural network is higher than that of the other two algorithms, i.e., SVM and BP. For example, after comparing 200 pieces of test data collected by a smartphone, the accuracy rates of the Bi-GRU neural network are 0.88%, 0.84%, and 0.89% for healthy, subhealthy, and unhealthy motion states, respectively, as shown in Figure 4. Similarly, the next higher performance was obtained by BP with 0.76%, 0.77%, and 0.75% for the three motion states, respectively. At the same time, the lowest recognition rates were observed in the case of the SVM classifier.

#### 4.2.2. Real-Time Recognition Test of the Proposed SHMS

In order to evaluate the prediction capability of the proposed system, the system was evaluated with real athlete data.  Figure 5 shows the recognition results of the sports training health status of the proposed SHMS. When the natural athlete data of an athlete with irregular lower limb gait were provided to the system, the system predicted the health status of the athlete as 0.02% healthy, 0.88 subhealthy, and 0.10% as unhealthy, which shows that the system is precise and accurate in predicting the health status of individuals.

## 5. Conclusion

The sports health status recognition method based on image processing can realize human health status without relying on fixed and complex medical equipment. This paper proposed a sports training health status recognition model based on the Bi-GRU neural network. This method employed smartphones for data collection and then developed a Bi-GRU neural network to build a neural network model. Furthermore, it combines deep learning technology and PyTorch deep learning platform to complete data collection and recognition of sports training health status. Finally, the motion data collected from an athlete have been used to assess the recognition performance of the system. Results showed that the proposed methodology could recognize the sports health status of individuals accurately.

## Figures and Tables

**Figure 1:** Schematic diagram of the athlete's thigh gait.

**Figure 2:** Unit structure of the GRU neural network.

**Figure 3:** Schematic diagram of the sports training health recognition model.

**Figure 4:** Histogram of comparison results.

**Figure 5:** Real-time recognition test of the proposed system.

**Table 1:** Performances of the machine learning algorithms.

Health type	Testing frequency	Recognition accuracy (%)		
		SVM	BP	Bi-GRU NN
Healthy	200	0.6225	0.7625	0.8814
Subhealthy	200	0.7541	0.7714	0.8475
Unhealthy	200	0.7285	0.7526	0.8936

## Data Availability

The data used to support the findings of this study are included within the article.

## References

[1] Xu Y., Guo X. (2020). Application of FPGA and complex embedded system in sports health data monitoring system. *Microprocessors and Microsystems*.

[2] Li S., Zhang B., Fei P., Shakeel P. M., Samuel R. D. J. (2020). Computational efficient wearable sensor network health monitoring system for sports athletics using IoT. *Aggression and Violent Behavior*.

[3] Xu Y., Jiang F., Du J., Gong D. (2019). A cross-domain collaborative filtering algorithm with expanding user and item features via the latent factor space of auxiliary domains. *Pattern Recognition*.

[4] Valchinov E., Antoniou A., Rotas K., Pallikarakis N. Wearable ECG system for health and sports monitoring.

[5] Alemayehu B., Warner K. E. (2004). The lifetime distribution of health care costs. *Health Services Research*.

[6] Xu Y., Chu Y., Jiang F., Guo Y., Gong D. (2018). SVMs classification based two-side cross domain collaborative filtering by inferring intrinsic user and item features. *Knowledge-Based Systems*.

[7] French E., Jones J. B. (2004). On the distribution and dynamics of health care costs. *Journal of Applied Econometrics*.

[8] Pinedo V. R., Westbury L. D., Syddall H. E. (2019). Health care costs associated with muscle weakness: a UK population-based estimate. *Calcified Tissue International*.

[9] Smith J. A., Braunack M. A., Wittert G., Warin M. (2008). “It’s sort of like being a detective”: understanding how Australian men self-monitor their health before seeking help. *BMC Health Services Research*.

[10] Boyes A., Newell S., Girgis A., McElduff P., Sanson F. R. (2006). Does routine assessment and real-time feedback improve cancer patients’ psychosocial well-being?. *European Journal of Cancer Care*.

[11] Liu L., Stroulia E., Nikolaidis I., Miguel C. A., Rios R. A. (2016). Smart homes and home health monitoring technologies for older adults: a systematic review. *International Journal of Medical Informatics*.

[12] Choi R., Hwang B. D., Hwang B. D. (2017). The relevance of socioeconomic class recognition and subjective health status of injured workers. *The Korean Journal of Health Service Management*.

[13] Xu Y., Yang J., Xie Z. (2014). Training SVMs on a bound vectors set based on Fisher projection. *Frontiers of Computer Science*.

[14] Park S. B. (2001). Recognition status of health-related to smoking, alcohol drinking, and stress in a work place. *Journal of the Korean Academy of Family Medicine*.

[15] Kim M. J., Lim Y. R., Kwak H. K. (2008). Dietary behaviors and body image recognition of college students according to the self-rated health condition. *Nutrition research and practice*.

[16] Ning X., Wang X., Xu S. (2021). A review of research on co‐training. *Concurrency and Computation: Practice and Experience*.

[17] Zhang J., Sun J., Wang J., Yu X. G. (2020). Visual object tracking based on residual network and cascaded correlation filters. *Journal of Ambient Intelligence and Humanized Computing*.

[18] Zhang X., Yang Y., Li Z., Ning X., Qin Y., Cai W. (2021). An improved encoder-decoder network based on strip pool method applied to segmentation of farmland vacancy field. *Entropy*.

[19] Zhang J., Liu Y., Liu H., Wang J. (2021). Learning local-global multiple correlation filters for robust visual tracking with kalman filter redetection. *Sensors*.

[20] Yu X., Zhan D., Liu L., Lv H., Xu L., Du J. (2021). A privacy-preserving cross-domain healthcare wearables recommendation algorithm based on domain-dependent and domain-independent feature fusion. *IEEE Journal of Biomedical and Health Informatics*.

[21] Huang Z., Zhang Y., Li Q. (2020). Joint analysis and weighted synthesis sparsity priors for simultaneous denoising and destriping optical remote sensing images. *IEEE Transactions on Geoscience and Remote Sensing*.

[22] Liu R., Ning X., Cai W., Li G. (2021). Multiscale dense cross-attention mechanism with covariance pooling for hyperspectral image scene classification. *Mobile Information Systems*.

[23] Zhang L., Wang X., Dong X., Sun L., Cai W., Ning X. (2021). Finger vein image enhancement based on guided tri-Gaussian filters. *ASP Transactions on Pattern Recognition and Intelligent Systems*.

[24] Mehta D. D., Zañartu M., Feng S. W., Cheyne H. A., Hillman R. E. (2012). Mobile voice health monitoring using a wearable accelerometer sensor and a smartphone platform. *IEEE Transactions on Biomedical Engineering*.

[25] Lee K. (2003). *Globalization and Health: An Introduction*.

[26] Foerster F., Smeja M., Fahrenberg J. (1999). Detection of posture and motion by accelerometry: a validation study in ambulatory monitoring. *Computers in Human Behavior*.

[27] Bao L., Intille S. S. Activity recognition from user-annotated acceleration data.

[28] Kwapisz J. R., Weiss G. M., Moore S. A. (2011). Activity recognition using cell phone accelerometers. *ACM SigKDD Explorations Newsletter*.

[29] Jiang W., Yin Z. Human activity recognition using wearable sensors by deep convolutional neural networks.

[30] Ronao C. A., Cho S.-B. (2016). Human activity recognition with smartphone sensors using deep learning neural networks. *Expert Systems with Applications*.

[31] Shafique M. A., Hato E. (2015). Use of acceleration data for transportation mode prediction. *Transportation*.

[32] Hochreiter S., Schmidhuber J. (1997). Long short-term memory. *Neural Computation*.

[33] Cho K., Van M. B., Gulcehre C. Learning phrase representations using RNN encoder-decoder for statistical machine translation.

[34] Frank A., Asuncion A. (2010). UCI machine learning repository.

[35] Zhang J., Wang W., Lu C., Wang J., Sangaiah A. K. (2020). Lightweight deep network for traffic sign classification. *Annals of Telecommunications*.

[36] Zhang Y., Li W., Zhang L., Ning X., Sun L., Lu Y. (2020). AGCNN: adaptive gabor convolutional neural networks with receptive fields for vein biometric recognition. *Concurrency and Computation: Practice and Experience*.

[37] Cai W., Wei Z. (2020). Remote sensing image classification based on a cross-attention mechanism and graph convolution. *IEEE Geoscience and Remote Sensing Letters*.

[38] Gu Y., Chen A., Zhang X., Fan C., Li K., Shen J. (2021). Deep learning based cell classification in imaging flow cytometer. *ASP Transactions on Pattern Recognition and Intelligent Systems*.

